# Schwannoma: A Rare Etiology of Pancoast Syndrome

This article has been retracted.

**DOI:** 10.7759/cureus.19418

**Published:** 2021-11-09

**Authors:** Fahad A Alshammari, Abdulmohsen M Alotaibi, Mahdi A Alali, Nawaf S Alkhileiwi, Sultan M Alshammari, Mansour T Albagami, Yasser G Alarimah, Faisal A Aldughaim, Kawther A Alsadady, Faisal F Alshammari, Kouther M Alhedires, Noor A Albejais, Mohammed F Alharbi, Awadh M Alharthi, Malak Alshammari

**Affiliations:** 1 Family Medicine, Imam Abdulrahman Bin Faisal University, Dammam, SAU; 2 Family Medicine, King Abdulaziz Hospital, Taif, SAU; 3 Family Medicine, King Faisal University, Hofuf, SAU; 4 Family Medicine, Umm Al-Qura University, Mecca, SAU; 5 Family Medicine, AlMaarefa University, Ad Diriyah, SAU; 6 Family Medicine, Dar Al Uloom University, Riyadh, SAU; 7 Family Medicine, University of Hail, Hail, SAU; 8 Family Medicine, Prince Saud Bin Jalawy Hospital, Al-Mubarraz, SAU; 9 Family Medicine, Qassim University, Qassim, SAU; 10 Family Medicine, King Faisal Hospital, Taif, SAU; 11 Internal Medicine, Imam Abdulrahman Bin Faisal University, Dammam, SAU

**Keywords:** case report, musculoskeletal disorders, schwannoma, rotator cuff pathology, shoulder pain

## Abstract

Musculoskeletal disorders represent a major public health problem and they are frequently managed in primary care centers. Shoulder pain is a frequent musculoskeletal complaint and it can result from intrinsic disorders of the shoulder or referred pain. We present the case of a 24-year-old woman who presented to the family medicine clinic complaining of left shoulder pain for three months duration. The pain was not associated with numbness or weakness. There was no history of preceding trauma. The initial diagnosis was supraspinatus tendinosis. The patient was prescribed oral analgesics and was advised to undergo multiple physiotherapy sessions. Later, the patient presented to the clinic again and reported she did not have any improvement in her symptoms. The patient was referred to the orthopedic clinic for further evaluation and management. The patient underwent a frontal radiograph of the chest which demonstrated a well-defined opacity located in the apex of the left lung. A computed tomography scan of the chest demonstrated the presence of erosion to the vertebral body raising the suspicion for a neurogenic tumor as was later supported by magnetic resonance imaging. The patient underwent video-assisted thoracotomy with brachial plexus exploration. Complete resection of the tumor was achieved with no complications. The present case highlights those common musculoskeletal complaints, such as shoulder pain, which could indicate underlying non-orthopedic pathology.

## Introduction

Musculoskeletal disorders represent a major public health problem and they are frequently managed in primary care centers. Shoulder pain is a frequent musculoskeletal complaint and it can result from intrinsic disorders of the shoulder joint or as referred pain due to another underlying pathology. A prospective study by Silverstein et al. [1] found that up to 20% of adults in the working population experienced shoulder pain over a one-year period. Intrinsic causes of shoulder pain include rotator cuff injury, tendinosis, impingement syndrome, frozen shoulder, osteoarthrosis, avascular necrosis, fractures, tumors, etc. [2]. However, shoulder pain can be a presentation of a more serious etiology, such as lung cancer [3]. Therefore, detailed history taking and appropriate physical examination should be conducted to identify any red-flag indicators. Imaging studies should be performed if the patient shows no clinical improvement after the trial of conservative and symptomatic measures. Here, we describe the case of a young woman who presented with chronic left shoulder pain that was initially managed as a rotator cuff injury. However, the patient was found to have schwannoma causing Pancoast syndrome.

## Case presentation

We present the case of a 24-year-old woman who presented to the family medicine clinic complaining of left shoulder pain for three months duration. The pain was stabbing in nature and was non-radiating. She reported that her shoulder pain was aggravated by raising her arms above her head. The pain was not associated with numbness or weakness. There was no history of preceding trauma. The patient scored the pain as 5 out of 10 on the severity scale. Further, the patient reported that the pain was constant with no progression in its severity. The past medical history was remarkable for intermittent asthma. She underwent laparoscopic appendectomy five years ago with no signs of complications. She did not require any previous hospitalization. She had never smoked nor consumed alcohol before. The family history was non-contributory.

Upon examination, the patient appeared comfortable. Her vital signs were within the normal limits. Examination of the left shoulder reveals a restricted range of motion of the left shoulder due to the pain. The supraspinatus impingement test was positive. However, examination of the right shoulder and the cervical spine revealed no abnormalities. Further, examination of other systems, including the cardiorespiratory and abdominal systems, was normal. Initial laboratory investigations, including hepatic and renal profiles, were within the normal limits (Table 1).

**Table 1:** Summary of the results of laboratory findings.

Laboratory Investigation	Unit	Result	Reference Range
Hemoglobin	g/dL	13.5	13.0–18.0
White Blood Cell	1000/mL	4.8	4.0–11.0
Platelet	1000/mL	370	140–450
Erythrocyte Sedimentation Rate	mm/hr.	11	0–20
C-Reactive Protein	mg/dL	3.8	0.3–10.0
Total Bilirubin	mg/dL	0.5	0.2–1.2
Albumin	g/dL	4.1	3.4–5.0
Alkaline Phosphatase	U/L	48	46–116
Gamma-glutamyltransferase	U/L	16	15–85
Alanine Transferase	U/L	18	14–63
Aspartate Transferase	U/L	20	15–37
Blood Urea Nitrogen	mg/dL	11	7–18
Creatinine	mg/dL	0.8	0.7–1.3
Sodium	mEq/L	136	136–145
Potassium	mEq/L	3.8	3.5–5.1
Chloride	mEq/L	102	98–107

In view of the aforementioned clinical findings, the initial diagnosis was supraspinatus tendinosis. The patient was prescribed oral analgesic medications and was advised to undergo a number of physiotherapy sessions. Six weeks later, the patient presented to the clinic again and reported she did not have any improvement in her symptoms. Hence, the patient underwent a local injection of corticosteroid in the supraspinatus region. However, the patient returned back after one month with the progression of her pain, and the pain became associated with numbness radiating to his arm. Of note, the patient had not had any plain radiographs performed in the primary care clinic.

In light of the lack of clinical improvement despite the multiple physiotherapy sessions and the corticosteroid therapy, the patient was referred to undergo an ultrasound examination of the shoulder. The ultrasound demonstrated intact rotator cuff tendons with no evidence of tendinopathy or discrete tears. The patient was referred to the orthopedic clinic for further evaluation and management.

The patient underwent a frontal radiograph of the chest which demonstrated a well-defined opacity located in the apex of the left lung. The opacity was at an acute angle with the lung (Figure 1). The differential diagnoses of this mass were very broad. The differential diagnoses included loculated effusion, hematoma, lipoma, fibroma, metastases, and mesothelioma. A computed tomography scan of the chest with intravenous contrast was performed for further characterization. The scan demonstrated the presence of erosion to the vertebral body (Figure 2). Such findings raised the suspicion of a neurogenic tumor. Subsequently, the patient underwent magnetic resonance imaging which re-demonstrated the contrast-enhanced lesion with its extension to the adjacent neural foramen (Figure 3). The radiological diagnosis was a neurogenic tumor. Subsequently, the patient underwent an ultrasound-guided biopsy and the histopathological examination of the obtained specimen was consistent with schwannoma.

**Figure 1:** Plain radiograph demonstrating a well-defined oval-shaped opacity in the apical zone of the left lung (arrow).

**Figure 2:** Coronal computed tomography image demonstrating a homogenous mass (arrow) in the left lung apex with erosion of the underlying vertebra (short arrow).

**Figure 3:** Magnetic resonance image demonstrating the mass lesion (arrow) with contrast-enhancement with extension to the neural foramen (short arrow).

The case was discussed in the multidisciplinary oncology team meeting to make the appropriate management plan for the patient. Resection of the tumor was planned and the patient agreed to proceed with the surgery. The patient underwent video-assisted thoracotomy with brachial plexus exploration. Complete resection of the tumor was achieved with no complications. The patient tolerated the procedure well and had an uneventful recovery. The patient was discharged on the sixth postoperative day. After two months of follow-up, the patient remained asymptomatic with no active complaints.

## Discussion

We present the case of a young woman with schwannoma, which is an unusual cause of Pancoast syndrome resulting in chronic shoulder pain. Pancoast syndrome is classically described with superior pulmonary sulcus tumor. Due to its apical pulmonary location, the tumor presents with clinical features resulting from an invasion to the brachial plexus or the stellate ganglion [4]. It is worth noting that chest X-ray is a valuable investigation in patients with suspected Pancoast tumor since it is normal in less than 2% of the cases [5]. Despite this, the diagnosis of Pancoast tumor is often delayed [6].

Schwannoma is a slow-growing tumor arising from the nerve sheath. Paravertebral thoracic schwannoma is a rare location. Schwannoma is often a solitary tumor and has a surrounding capsule [7]. Schwannoma can develop at any age group and there is no sex predilection. It is more common to arise in the extremities followed by the head and neck areas [8]. As in the present case, schwannoma may arise from the posterior mediastinum.

Considering its benign nature and slow growth behavior, the tumor is usually asymptomatic. Neurological symptoms develop when the tumor grows to a large size [9]. The clinical manifestation of schwannoma in the present case was unique. The patient had chronic shoulder pain for several months that was mimicking a rotator cuff injury. This emphasizes the importance of not delaying the medical imaging if indicated.

Regarding the radiological findings, schwannoma appears as a well-defined mass lesion that displaces but does not invade the surrounding structures [8]. While fatty and cystic degenerations are common, calcification is an unusual feature for schwannoma [10]. Computed tomography scan is inferior to magnetic resonance imaging in the accuracy for the diagnosis of schwannoma, but it is often performed first, as in the present case [10]. The computed tomography scan can demonstrate intense contrast enhancement of the lesion with the remodeling of the surrounding bone. Lastly, magnetic resonance imaging has a characteristic manifestation for schwannoma with low signal intensity in the T1-weighted image, high signal intensity in the T2-weighted image, and intense contrast enhancement [11].

## Conclusions

The present case highlights the fact that common musculoskeletal complaints, such as shoulder pain, could indicate underlying non-orthopedic pathology. Physicians should keep a high index of suspicion for malignancy in patients with shoulder pain who have unusual responses to the appropriate conservative management. The case also demonstrates that schwannoma could be a mimicker of rotator cuff injury causing a delay in the diagnosis and management. Hence, primary care physicians should not be reluctant in requesting imaging investigations, such as plain radiographs, if indicated.
